The article "Hemophagocytic Lymphohistiocytosis Secondary to Disseminated Histoplasmosis in AIDS Patient" was published in 2021. Journal: Cureus.

# Hemophagocytic Lymphohistiocytosis Secondary to Disseminated Histoplasmosis in AIDS Patient

**DOI:** 10.7759/cureus.20347

**Published:** 2021-12-11

**Authors:** Raed Atiyat, Riyashat Kazmi, Krunal Trivedi, Hamid S Shaaban

**Affiliations:** 1 Medical Education, Saint Michael's Medical Center, Newark, USA; 2 Hematology and Oncology, Saint Michael's Medical Center, Newark, USA

**Keywords:** differential for fever of unknown origin, immunocompromised patient, disseminated histoplasmosis, hiv aids, hemophagocytic lymphohistiocytosis (hlh)

## Abstract

Hemophagocytic lymphohistiocytosis (HLH) is a rare and life-threatening syndrome that is often underdiagnosed. There are limited treatments and clinical outcomes documented in adults, more so in the immunocompromised population. Here, we described the clinical features, diagnosis, treatment, and clinical outcome of an HLH secondary to histoplasmosis in an AIDS patient.

## Introduction

Hemophagocytic lymphohistiocytosis (HLH) is a disorder that occurs due to hemophagocytosis and systemic hyperactivation of the immune system that often leads to inflammatory cytokine overproduction. HLH is a clinical entity that can be inherited or due to secondary causes such as infections, autoimmune disorders, immunosuppression, and malignancy.

Secondary (acquired) HLH, is a rather aggressive illness that demands timely identification and rapid commencement of proper management [1]. While protocols include inclusion criteria, they are mainly used and accepted for diagnosing [2]. This urgency however is stymied by controversial management strategies. Management of HLH secondary to disseminated histoplasmosis is poorly delineated and decisions regarding timing to initiate immunosuppressive therapy as per HLH 2004 standards are greatly questioned [3]. While illness due to *Histoplasma capsulatum* can initially present symptomless, it can quickly develop to a critical disease with hematogenous spread, which a previous study revelated occurred in 0.05% out of 2000 patients, more so in elderly and immunocompromised individuals [4]. Due to nonspecific generalized symptoms, HLH manifesting in the setting of an initial diagnosis of sepsis can often miss and underdiagnose HLH. This often delays the diagnosis of HLH and its appropriate therapy. Herein, we present a case of a 55-year-old immunocompromised male who developed histoplasmosis-induced HLH.

## Case presentation

A 55-year-old male with a past medical history of uncontrolled acquired immunodeficiency syndrome (AIDS), type 2 diabetes mellitus, hypertension, hyperlipidemia, coronary artery disease, hypothyroidism, pancytopenia, gastric bypass presented to the emergency department complaining of fatigue, fever, chills, diarrhea, dysuria, urinary retention, dyspnea on exertion, palpitations, cough with productive white sputum, and recent 20-pound weight loss. He denied chest pain, orthopnea, wheezing, or lower extremity edema.

The article "Hemophagocytic Lymphohistiocytosis Secondary to Disseminated Histoplasmosis in AIDS Patient" was published in 2021. Journal: Cureus.

On presentation, the patient was tachycardiac, febrile (101.3°F), normal respiratory rate, saturating well on room air, and with stable blood pressure. Physical examination was remarkable for dry oral mucosa, conjunctival pallor, cachexia, rales of the right lung field, tachycardia, and hepatosplenomegaly. The patient’s laboratory results included complete blood count (CBC; Table 1), comprehensive metabolic panel (CMP; Table 2), iron panel (Table 3), and inflammatory markers (Table 4). The patient’s natural killer (NK) cell count was too low to get a numeric result. The laboratory values below helped guide the diagnosis. 

**Table 1:** Complete blood count

Complete blood count	Result	Reference range
White blood cell	1.70	4.4-11.00
Red blood cell (10^6^/uL)	3.36	4.32-5.72
Hemoglobin (g/dL)	9.4	13.5-17.5
Hematocrit (%)	28.0	38.8-50.0
Mean corpuscular volume (fL)	83.3	81.2-95.1
Mean corpuscular hemoglobin (pg)	27.9	27.5-33.2
Mean corpuscular hemoglobin concentration (g/dL)	33.5	33.4-35.5
Red cell distribution width (%)	19.4	11.8-15.6
Platelets (10^3^/uL)	14	150-450
Mean platelet volume (fL)	13.1	7.4-11.0
Manual differential		
Neutrophils	87	
Bands (relatives)	6	
Lymphocytes (relatives)	7	
Monocytes (relatives)	4	
Neutrophils (absolute)	1.5	1.7-7.0 × 10^3^/uL
Bands (absolute)	0.2	
Lymphocytes (absolute)	0.1	0.9-2.9 × 10^3^/uL
Monocytes (absolute)	0.1	0.3-0.9 × 10^3^/uL
Vacuolated neutrophils	Rare	
Anisocytosis	Few (2+)	Rare, slight present
Burr cells	Moderate (3+)	
Ovalocytes	Few (2+)	
Dacrocytes	Few (2+)	

**Table 2:** Comprehensive metabolic panel

Comprehensive metabolic panel	Result	Reference range
Sodium	127	136-145 mmol/L
Potassium	5	3.5-5.3 mmol/L
Chloride	102	98-110 mmol/L
Bicarbonate	12	20-31 mmol/L
Anion gap	13	5-15 mmol/L
Blood urea nitrogen	43.0	6-24 mg/dL
Creatinine, serum	2.3	0.6-1.2 mg/dL
Glucose	75	70-140 mg/dL
Aspartate transaminase	121	10-36 u/L
Alanine aminotransferase	30	9-46 u/L
Alkaline phosphatase	308	40-115 U/L
Total protein	4.9	6.4-8.4 g/dL
Albumin	1.4	3.6-5.1 g/dL
Total bilirubin	3.8	0.2-1.2 mg/dL
Magnesium	1.9	1.5-2.5 mg/dL
Phosphorus	4.3	2.1-4.3 mg/dL
Bilirubin, direct	3.22	0.00-0.30 mg/dL
Calcium	6.6	8.6-10.4 mg/dL
Fibrinogen	135	200-393 mg/dL
Triglyceride	291	0-150 mg/dL

**Table 3:** Iron profile

Iron profile	Result	Reference range
Iron	34	50 150 ug/dL
Ferritin	>40,000	24-336 ng/ml
Total iron-binding capacity	100	250-400 ug/dL

**Table 4:** Inflammatory markers

Inflammatory markers	Result	Reference range
Ferritin	>40,000	24-336 ng/mL
Lactate dehydrogenase	683	122-222 u/L
Triglyceride	291	0-150 mg/dL
C-reactive protein	13.3	0.0-0.8 mg/dL
Procalcitonin	26.12	0.00-0.50 ng/mL
Erythrocyte sedimentation rate	72	0-30 mm/h
D-dimer	8598	0.0-500 ng/mL

When compared to the previous imaging weeks prior to Figure 1a, chest x-ray was suggestive of subpulmonic bilateral effusion as seen in Figure 1b. A computed tomography scan of the chest, abdomen, and pelvis was noted to have small bilateral effusion and trace ascites, diffuse interstitial lung markings, and patchy ground-glass consolidation in the posterior right upper lobe. The asterisks in Figure 2 highlights bilateral effusion, while the arrows in Figure 2 and Figure 3 highlight the patchy ground-glass appearance. A differential of pulmonary edema versus atypical pneumonia versus lymphangitic carcinomatosis was made as per imaging. In addition, there was a notable single 3.1 x 1.9 cm right retroperitoneal lymph node. In addition, MRI of the abdomen was obtained with and without contrast was suggestive of hepatomegaly, ascites, and deep mesenteric and retroperitoneal lymphadenopathy measuring 2.5 x 1.5 cm of indeterminate significance. Reticulin stain showed a nonspecific moderate increase in reticulin fibers seen within the hypercellular bone marrow areas. Iron stain displayed focal mild stainable iron deposits. Findings were characterized as nonspecific for HLH, however, may be associated with a myeloproliferative and/or myelodysplastic disorder, infectious process, reactive process.

The article "Hemophagocytic Lymphohistiocytosis Secondary to Disseminated Histoplasmosis in AIDS Patient" was published in 2021. Journal: Cureus.

**Figure 1:** (A) Chest x-ray from the previous admission displays no abnormalities; (B) chest x-ray displays subpulmonic effusions near diaphragm area, and the asterisks display increased congestion and infiltrate

**Figure 2:** CT scan of chest arrow displaying ground-glass consolidation, asterisks highlighting bilateral effusions

**Figure 3:** CT scan of the chest revealing patch ground-glass consolidation

Based on the HLH diagnostic criteria seen in Table 5, the patient had five out of eight criteria making the diagnosis for HLH very likely [5]. Also of note, hemophagocytosis score (HScore) for reactive hemophagocytic syndrome entails adding points based on Table 6 to give us a probability of diagnosing HLH [6]. Our patient was immunosuppressed (18 points), and had a fever of 101.3°F (33 points), hepatomegaly (23 points), cytopenia of three lineages (34 points), ferritin (50 points), triglyceride (44 points), fibrinogen (30 points), aspartate aminotransferase (30 points), and bone marrow features of HLH (0 points). Based on the HScore for reactive hemophagocytic syndrome, this patient has a score of 251 points with a >99% probability of hemophagocytic syndrome. An optimal cutoff is 169 points which accurately identifies 90% of patients.

The article "Hemophagocytic Lymphohistiocytosis Secondary to Disseminated Histoplasmosis in AIDS Patient" was published in 2021. Journal: Cureus.

**Table 5:** Hemophagocytic lymphohistiocytosis diagnostic criteria ^a^Hemoglobin <9 g/dL, platelets <100 x 10^9^/L, and neutrophils <1.0 x 10^9^/L ^b^Triglyceride ≥265 mg/dL and fibrinogen ≤150 mg/dL ^c^≥500 mg/L ^d^CD25 ≥2400 U/mL HLH: hemophagocytic lymphohistiocytosis; NK: natural killer; CD: cluster of differentiation

Molecular diagnosis consistent with HLH or presence of 5 out of 8 below diagnostic criteria
Fever
Splenomegaly
Cytopenia^a^ affecting ≥ 2 lineage
Hypertriglyceridemia and or hypofibrinogenemia^b^
Hemophagocytosis in bone marrow, spleen, or lymph node
Low or absent NK cell activity
Ferritin^c^
Soluble^d^

**Table 6:** HScore for reactive hemophagocytic syndrome, numerical value within the parenthesis are to be added in order to give cumulative number and help calculate the probability of HLH diagnosis ^a^Hemoglobin ≤9.2 g/dL, platelets ≤110,000/mm^3^, and WBC ≤5000/mm^3^ HScore: hemophagocytosis score; HLH: hemophagocytic lymphohistiocytosis; WBC: white blood cell

HScore for reactive hemophagocytic syndrome			
Hemophagocytosis in bone marrow	Yes (+35)	No (0)	
Known immunosuppression	Yes (+18)	No (0)	
Fever (F)	>102.9 (+49)	101.1-102.9 (+33)	<101.1 (0)
Organomegaly	Hepatomegaly and splenomegaly (+38)	Hepatomegaly or splenomegaly (+23)	No (0)
Cytopenia^a^	3 lineages (+34)	2 lineages (+24)	1 lineage (0)
Ferritin (ng/mL)	>6000 (+50)	2000-6000 (+35)	<2000 (0)
Triglycerides (mg/dL)	>354 (+64)	132.7-354 (+44)	<132.7 (0)
Fibrinogen (mg/dL)	≤250 (+30)	>250 (0)	
Aspartate aminotransferase (U/L)	≥30 (+19)	<30 (0)	

The patient was admitted to the intensive care unit and over the course of stay, he received atovaquone, vancomycin, azithromycin, levofloxacin, metronidazole, and IV hydrocortisone 100 mg three times daily as well as IV fluids as per sepsis fluid resuscitation. Cluster of differentiation (CD)4 and CD8 count done a year prior revealed CD4 44 (560-2700 x 10^3^/uL), CD8 61.48% (12-38%), CD4 helper T cell 7.87% (27-60%), viral load of 930,000. The patient was started on daily tbo-filgrastim, desmopressin (DDAVP) to address uremic-platelet dysfunction, and one dose of IVIG to address thrombocytopenia. Zithromax and Levaquin were both discontinued after acid-fast bacillus (AFB) results came back negative and he subsequently received IV daptomycin every 48 hours for vancomycin-resistant *Enterococcus faecium* (VRE) bacteremia. On day 5, both histoplasma antigen results were positive >15 ng/mL (reference range: <0.5 ng/mL) and Fungitell serum was >189 pg/mL (reference range: <80 pg/mL). The patient’s mental status was deteriorating and he developed widespread purpura with severe thrombocytopenia of 11 (reference range: 150-450 g/dL). At this point, a family discussion was held regarding goals of care, and the family expressed that the patient would have requested non-aggressive treatment. Unfortunately, the patient passed away shortly after.

The article "Hemophagocytic Lymphohistiocytosis Secondary to Disseminated Histoplasmosis in AIDS Patient" was published in 2021. Journal: Cureus.

## Discussion

Hemophagocytic lymphohistiocytosis (HLH) is a severe life-threatening syndrome of hyper inflammation often leading to multiorgan failure. Patients often present initially with sepsis in conjunction with high rates of mortality by the time HLH is diagnosed, at which point treatment has been already delayed. In untreated patients, mortality is 100%, thus early diagnosis and treatment are essential [1]. A status of AIDS with CD4 count < 200 cells per uL as seen in our patient bears a grim prognosis [1]. A common presentation noted in most cases is “fever of unknown origin.” Fever in an AIDS patient generates an exhaustive list of differential diagnoses that warrants extensive diagnostic workup, consultation, and testing. In addition, the identification of disseminated histoplasmosis can easily become overshadowed by other considerations such as opportunistic infections and tuberculosis and pneumocystis pneumonia (PCP). The difficulty in diagnosing both HLH and disseminated histoplasmosis is what makes this case rather challenging. Since early diagnosis and initiation of antifungal therapy appear to have a significant impact on the outcome, physicians should proceed cautiously, and meticulously explore histoplasmosis and HLH in cases of fever of unknown origin in an AIDS patient. By maintaining a preemptive strategy, the serum ferritin level, fibrinogen, triglycerides, microbiological test for histoplasmosis, and biopsies to determine yeast or hemophagocytosis can be ordered sooner [7]. Hemophagocytosis itself may not be an uncommon finding in AIDS either, as demonstrated by an autopsy case series of 56 patients, of whom 96% had AIDS and 20% had histological evidence of hemophagocytosis [8]. We also bring our attention to the dichotomy of sepsis being a common issue and HLH being a rare occurrence, yet we note the overlapping presence of hemophagocytosis described in patients with severe sepsis and multiple organ dysfunction syndrome [9]. Of 107, 64.5% autopsies of critically ill patients had hemophagocytosis in bone marrows biopsy [10]. The overlap of clinical and laboratory features between sepsis, AIDS, and HLH raises the dilemma of identifying HLH in AIDS patients. This certainly leads to HLH being significantly underdiagnosed in the AIDS population. 

As per HLH-2004 guidelines, the standard of care for severe or relapsing HLH is currently chemotherapy and transplantation of bone marrow [11,12]. Previously documented literature stated 10 out of 22 cases of HLH secondary to histoplasmosis who received amphotericin B survived, while at the same time three out of four patients treated with IVIG expired [4]. This indicates that treating the underlying cause of the disorder in a timely manner can eliminate the necessity of chemotherapy or bone marrow transplantation [1].

The article "Hemophagocytic Lymphohistiocytosis Secondary to Disseminated Histoplasmosis in AIDS Patient" was published in 2021. Journal: Cureus.

While there is no definitive diagnosis or golden confirmatory test available till this day, using multiple criteria, as many overlap, can strengthen the argument for diagnosis of HLH. It is imperative to identify the cause of the disorder, and treatment should not be delayed. A prime example of this is HIV-induced secondary HLH, when highly active antiretroviral therapy (HAART) therapy was initiated in these individuals, effective recovery was documented [13,14]. While Epstein Bar virus (EBV) induced secondary HLH required only immunosuppressive treatment [4], other infections required treating underlying cause with antimicrobials only in order to help resolve HLH [1].

## Conclusions

While there are many causes of HLH, we must find the optimal treatment and treat the underlying cause. While symptoms can be vague in nature, early diagnosis and management are imperative for patient’s survival as previously discussed. This case demonstrated the importance of considering histoplasmosis as the cause of HLH in the adult population, especially immunocompromised patients.
